# Development of microporous activated Aloji clay for adsorption of lead (II) ions from aqueous solution

**DOI:** 10.1016/j.heliyon.2019.e02799

**Published:** 2019-11-20

**Authors:** K.S. Obayomi, M. Auta

**Affiliations:** a Chemical Engineering Department, Landmark University, PMB 1001 Omu- Aran, Kwara State, Nigeria; b Chemical Engineering Department, Federal University of Technology, PMB 65, Minna, Niger State, Nigeria

**Keywords:** Environmental science, Materials chemistry, Thermodynamics, Kinetics, Adsorption, Optimization, Aloji clay, Adsorption isotherm

## Abstract

Aloji clay was activated with HCl at optimal conditions variables (acid concentration, activation temperature and time) using central composite design with yield (%) and Pb^2+^ uptake as responses targeted. The obtained optimum conditions for high yield (%) and Pb^2+^ uptake were at 0.5 M, 100 °C and 120 min. At these conditions, BET surface area of 214.80 m^2^/g of the microporous activated adsorbent gave a maximum monolayer of 333.33 mg/g for Pb^2+^. The effects of equilibrium time, initial Pb^2+^ concentration, temperature and adsorbent dosage were examined. Pseudo-second-order kinetic and Freundlich models best described Pb^2+^ adsorption onto Aloji activated clay as compared to the other isotherms and kinetics models investigated. The adsorption process was spontaneous, exothermic and physical as revealed by the nature of the thermodynamic studies. The study shows that the discharge of harmful substances posed by industrials into water bodies can be salvage by effective and efficient use of activated Aloji clay.

## 1 Introduction

Rapid massive industrialization in the last decades has been accompanied with emergence of new pollutants posing serious health and environmental global challenges. One of the greatest ecological challenge making difficult issues to living creatures is water pollution. The expulsion of these different poisonous substances from water and wastewater bodies has been a principal interest of numerous researchers and scientists worldwide [1, 2, 3].

Water containing heavy metals have been researcher's major concern over the years because of their lethality to human being, environment and aquatic life. However, because they do not degrade organically (natural pollutant) their presence in water bodies and industrial effluent is a severe challenge to human health. Lead is a toxic metal that damages human nervous structure and causes brain ailment. Furthermore, lengthy span introduction to lead may cause nephropathy, abdominal torments and a lady's capacity to produce [4]. Procedures such as technologies of membrane filtration, reverse osmosis chemical precipitation, ion exchange, evaporation, solvent extraction, ion exchange and electrochemical treatment, have been employed severally to eliminate these harmful toxins from wastewater. Because of the inability of these methods to adsorb metals with low concentration, the use of adsorption has been employed which has proven to be effective and efficient because of its reduced cost and ease of handling [5, 6, 7].

The selection of an adsorbent depends favorably on certain factors which are use of operation, material cost, adsorption capacity, reuse potential and its ability to be regenerated after use [8].

Several agricultural materials of wide availability have been explored in different form as adsorbents for pollutants elimination from wastewater [9, 10, 11, 12]. Great attention has now developed towards naturally occurring adsorbents but ideally with high adsorption capacity for expelling poisons from sullied waters. Though, different adsorbents have been used for the treatment of these wastewater but naturally accessible clays have been the adsorbents of choice [10, 13, 14, 15].

Efficient and effective crude and altered (modified) clays for purpose of adsorption have been broadly utilized. The fact that new difficulties of contamination issues continues surfacing, calls has now being made for a consistent research findings towards an effective, less expensive and progressively productive solution for the problems [16, 17]. Clay treatment with acids has been established to be the best and most effective change amid numerous approaches. Acid treatments help in specific surface area increase, acidic centers, surface functional group modification and high porosity with solids [18]. The most wide used in acid treatment of clays are HCl and H_2_SO_4_ acids among others since they show solid warmth by the process variable and incredible outcomes in adsorption capacity, porosity and specific surface area [19]. This investigation is aimed at studying the probable utilization of natural rich local clay as an absorbent in aqueous solution for Pb^2+^ adsorption.

## 2 Materials and method

### 2.1 Materials

Pb(NO_3_)_2_ and HCl were acquired from Sigma- Aldrich chemicals. The parent clay used was gotten from Aloji in Ofu local government of Kogi state, Nigeria; which was crushed, grounded, sieved to size particle of 125 μm and dried for 2h in an oven at 105 °C.

### 2.2 Stock solution preparation

A known quantity of Pb (NO_3_)_2_ was dissolved in 1000 mL of distilled water so as to prepare Pb^2+^ stock solution. Other concentrations ranging from 30, 60, 100 and 150 mg/L were by serial dilution prepared from the stock solution and for each experiment freshly prepared solution was used.

### 2.3 Design of experiment using central composite design (CCD)

CCD was used for the optimization of Aloji clay modification using the selected activation variables; acid concentration, activation time and temperature. The optimization responses of this process were Pb^2+^ uptake and percentage yield. The empirical model using optimal predictor cubic equation was used to correlate the variables and responses as given by Eq. (1).

(1) $$Y=\beta_{0\;}+\overset{n}{\underset{i=1}{\sum }}\beta_{i}x_{i}+{\left(\overset{n}{\underset{i=1}{\sum }}\beta_{ii}x_{i}\right)}^{2}+{\left(\overset{n}{\underset{i=1}{\sum }}\beta_{iii}x_{i}\right)}^{3}+\overset{n-1}{\underset{i=1}{\sum }}\overset{n}{\underset{j=i+1}{\sum }}\overset{n+1}{\underset{k=i+j+1}{\sum }}\beta_{ijk}x_{i}x_{j}x_{k}$$

Y = response foreseen, β_0_ = coefficient constant, βiii = coefficient constants, βijk = interaction coefficients while xi, xj and xk are the parameters of the coded values considered. CCD are categorized by three operations which is: axial runs (2n), factorial runs (2^n^) and center runs which translated into axial points (6), factorial points (8) and the centre point replicates (6) translating into 20 experimental runs as generated by the Design Expert software (statistical) version 7.0.0. The coded levels and their values corresponding are depicted in Table 1.

**Table 1:** Independent parameters and their coded levels.

Parameters (Factors)	Code	Unit	Variable levels (coded)		
			-1	0	+1
Acid concentration	x_1_	M	0.50	2.25	4.0
Activation temperature	x_2_	°C	70.0	85.0	100.0
Time of activation	x_3_	min	30.0	75.0	120.0

### 2.4 Preparation of clay adsorbent

The following factors for optimization are considered: acid concentration (0.5–4 M), activation temperature (70–100 °C) and activation time (30–120 min) was used to activate the dried Aloji clay. 10 g of the raw clay was weighed into a 250 mL beaker and 50 mL of 0.5 M HCl solution was added and positioned on a magnetic hotplate stirrer. The set temperature of the mixture was at 70 °C and mixed energetically for 30 min at 140 rpm. At the end of the experiment, the activated acid clay was washed with water (distilled) to ensure the supernatant achieve neutrality (pH 6.9), thereafter the clay was oven dried at 120 °C for 3 h and was later stored in a flask for additional use. The same procedure was repeated for others as generated by the experimental design (DOE) in Table 2.

**Table 2:** Aloji clay activation using experimental design matrix (RSM).

Runs	X_1_ (M)	X_2_ (^0^ C)	X_3_ (min)	Yield (%)	Pb^2+^ (%) removal
1	-1	-1	-1	64.10	95.33
2	+1	-1	-1	64.80	93.44
3	-1	+1	-1	61.77	93.89
4	+1	+1	-1	58.40	92.67
5	-1	-1	+1	58.20	93.16
6	+1	-1	+1	57.50	92.22
**7**	**-1**	**+1**	**+1**	**55.65**	**97.33**
8	+1	+1	+1	65.13	92.56
9	-1	0	0	63.13	95.78
10	+1	0	0	60.32	93.22
11	0	-1	0	64.77	95.33
12	0	+1	0	60.60	94.67
13	0	0	-1	60.30	93.67
14	0	0	+1	63.50	96.33
15	0	0	0	61.28	96.67
16	0	0	0	62.83	96.22
17	0	0	0	63.50	95.44
18	0	0	0	62.50	95.56
19	0	0	0	61.70	95.67
20	0	0	0	62.20	95.89

x_1_ = Acid concentration, x_2_ = temperature, x_3_ = Activation time.

The dependability of the analysis completed by the ANOVA was estimated by the responses unpredictability values which was expressed by determination coefficient R^2^, the Fisher's test and likelihood P-value (95% level of certainty). The percentage yield response of the Aloji clay after subjection to acid activation, washing and drying was determined using Eq. (2).

(2) $$\left(\%\right)Yield=\frac{\text{ ​Dried ​clay ​after ​activation ​in ​grams}}{\text{ ​Dried ​clay ​before ​activation ​in ​grams}}\times 100$$

0.1 g of activated Aloji clay was positioned in a 250 mL set of conical flasks containing 100 mL of Pb^2+^ (100 mg/L) concentration in a typical batch experiment as the Pb^2+^ initial pH was maintained. The flasks at 30 °C were positioned on an isothermal shaker with 140 rpm attuned shaker speed. After 1 h, the residual Pb^2+^ concentration was measured using Atomic Absorption Spectroscopy (Perkin Elmer, Model A Analyst 200). The percentage of Pb^2+^ removal was calculated using Eq. (3)

(3) $$Pb^{2+}+\text{ ​}removal\;\left(\%\right)=\frac{Initial\;Pb^{2+}\;concentration\;–Final\;Pb^{2+}concentration}{Intial\;Pb^{2+}concentration}\times 100$$

The optimum condition for run 7 was selected, characterized and used for further batch adsorption studies.

### 2.5 Aloji clay characterization

The analyses that were carried out on the Aloji clay before and after activation are elemental composition using X-Ray Fluorescence (XRF) (Model-PW2400 of Phillips), surface chemistry using Fourier Transform Infrared Spectroscopy (FT-IR) (Perkin-Elmer infrared spectrophotometer) and the surface area using Brunauer Emmett Teller (BET) (Micrometrics ASAP 2020).

### 2.6 Batch equilibrium and kinetics studies

The equilibrium batch adsorption were studied using a set of conical flasks (250 mL) comprising 100 mL of Pb^2+^ at several concentrations of 30, 60, 100 and 150 mg/L. The activated Aloji clay adsorbent of 0.1 g (125 μm) was then added and immediately placed on shaker (isothermal) set at 30 °C for 2 h and 140 rpm shaker speed to achieve equilibrium. At different interval of time, adsorbate samples were taken, filtered and measured so as to determine the remaining concentration in the solution until equilibrium is attained using Atomic Absorption Spectroscopy (AAS). Subsequently, the shaker (isothermal) temperature was attuned to 40 °C and 50 °C respectively and the experimental process was repeated. At equilibrium, Pb^2+^ amount adsorbed q_e_ (mg/g) at time t; was determined by Eq. (4):

(4) $$q_{e}=\frac{\left({\text{C}}_{\text{o ​}-\text{ ​}}{\text{C}}_{\text{e}}\text{ ​}\right)\text{V}}{\text{w}}$$

Where C_o_ and C_e_ (mg/L) are initial and equilibrium concentration of the Pb^2+^, respectively; V (L) is the volume of the solution; and W (g) is the adsorbent mass.

## 3 Results and discussion

### 3.1 XRF analysis

The Aloji clay elemental composition was determined by XRF analysis and the outcome is depicted in Table 3. The parent clay major constituents are alumina and silica though other elements such as Fe, K, Ti, Ca and Mg were also observed at varied composition. Loss on Ignition (LOI) demonstrates level of unpredictable substance in form of organic material (plant debris) as contained in the sourced clay. The introduction of this organic material might be outlined down to the clay's source due to the deterioration of plants and animals. The LOI value of 15.0 % is higher than the value reported by [20] and this could be an effect of the geographical location where the clay sample was sourced.

**Table 3:** Elemental composition of raw Aloji clay.

Elemental Composition	Weight (%)
SiO_2_	53.92
Al_2_O_3_	27.22
Fe_2_O_3_	0.94
K_2_O	1.24
TiO_2_	0.22
CaO	0.61
MgO	0.42
LOI	15.0

### 3.2 Response surface methodology design of experiment

CCD was used to carry out the polynomial regression development equations for the correlation analysis between the percentage yield and its Pb^2+^ uptake ability. Eqs. (5) and (6) give the final coded variables empirical models (exclusion of insignificant terms) for the yield and Pb^2+^ uptake on the adsorbent respectively. The relative predictor power R^2^ which gives the quality of the model was within the desirability range of 0.9726 (yield) and 0.9627 (Pb^2+^ removal). These values relative high nature is a demonstration that good relationship exist between the experimented and the predicted values gotten for the optimized parameters (acid concentration, activation temperature and time) under study.

(5) Y _HCL_ = 62.47–1.41x_1_ – 2.08x_2_ + 1.60x_3_ + 0.76x_1_x_2_ + 1.43x_1_x_3_ + 1.73x_2_x_3_ – 0.95x_1_^2^ – 0.0059x_2_^2^ – 0.78x_3_^2^ + 1.78x_1_x_2_x_3_ + 1.63x_1_^2^x_2_ – 3.17x_1_^2^x_3_ + 2.17x_1_x_2_^2^

(6) R _HCL_ = 95.74–1.28x_1_ – 0.33x_2_ + 1.33x_3_ – 0.39x_1_x_2_ – 0.32x_1_x_2_ + 0.84x_2_x_3_ – 0.99x_1_^2^ – 0.49x_2_^2^ – 0.49x_3_^2^ – 0.56x_1_x_2_x_3_ + 0.62x_1_^2^x_2_ – 1.34x_1_^2^x_3_ + 0.18x_1_x_2_^2^

Result on Table 1 shows the percentage removal for Pb^2+^ was in the range of 92.22–97.33 % and the yield range (%) was 55.65–65.13 % respectively. These results can be seen on the total experimental design matrix and their responses as depicted in Table 1. Cubic models for the two responses as choosen by the design expert software based on the highest order polynomial were used and going by the sequential sum of square, the models were not aliased and the additional terms were significant. The center points (15–20 runs) were carried out in order to check data experimental error and reproducibility. Based on the result in Table 1, run 7 gave the highest percentage of Pb^2+^ at an optimum conditions of 0.5 M, 120 min and 100 °C and as a result it was mass produced, characterized and used further to determine the effects of pH, adsorbent dosage, initial Pb^2+^ concentration, adsorption equilibrium, kinetic and thermodynamic studies.

### 3.3 Analysis of variance (ANOVA)

Cubic models as suggested by the central composite design (CCD) as shown in Tables 4 and 5 were generated for percentage yield and Pb^2+^ uptake. The cubic models accuracy and their significant on the both responses were further emphasized using the ANOVA. The surface cubic models response of the ANOVA mean square was gotten by dividing sum of squares, error variance and the model by their individual degree of freedom [21]. The F- value and Prob > F variance fishers ratio for the activated Aloji clay yield model were 16.38 and 0.0013. The yield percentage showed that significant model terms are x_1_, x_2_, x_3,_ x_1_x_2,_ x_2_x_3_, x_1_x_3_ x_1_x_2_x_3,_ x_1_^2^ × _2_, x_1_^2^ × _3_ and x_1_x_2_^2^ while x_1_^2^, x_2_^2^, and x_3_^2^ are insignificant. The regression coefficient value of R^2^ of 0.97 indicates the existence of good relationship between the predicated and the experimental data (Fig. not shown). F-value and Prob > F of 11.90 and 0.003 respectively, were obtained for Pb^2+^ uptake model. The model Pb^2+^ removal by activated Aloji clay showed significant terms at x_1_, x_3,_ x_2_x_3_, x_1_^2^, x_1_x_2_x_3,_ and x_1_^2^ × _3_. Also, a good relationship between the experimental and the predicted data was seen to have existed judging from the coefficient R^2^ value of 0.96 (Fig. not seen).

**Table 4:** Response surface ANOVA cubic model on yield for Aloji clay activation.

Source	Sum of square	Degree of freedom	Mean square	F- value	Prob > F
Model	126.170	13	9.710	16.380	0.0013
x_1_	3.950	1	3.950	6.660	0.0417
x_2_	8.690	1	8.690	14.680	0.0087
x_3_	5.120	1	5.120	8.640	0.0260
x_1_x_2_	4.670	1	4.670	7.880	0.0309
x_1_x_3_	16.390	1	16.390	27.660	0.0019
x_2_x_3_	23.840	1	23.840	40.240	0.0007
x_1_^2^	2.500	1	2.500	4.230	0.0856
x_2_^2^	9.6E-005	1	9.6E-005	1.6E-004	0.9903
x_3_^2^	1.670	1	1.670	2.820	0.1442
x_1_x_2_x_3_	25.380	1	25.380	42.840	0.0006
x_1_^2^ x_2_	4.240	1	4.240	7.160	0.0367
x_1_^2^ x_3_	16.120	1	16.120	27.200	0.0020
x_1_x_2_^2^	7.530	1	7.530	12.700	0.0119
Residual	3.550	6	0.590	-	-
Lack of fit	0.390	1	0.390	0.620	0.4676
Pure error	3.160	5	0.630	-	-

**Table 5:** Response surface ANOVA cubic model forPb^2+^ removal by activated Aloji clay.

Source	Sum of square	Degree of freedom	Mean square	F- Value	Prob > F
Model	42.390	13	3.260	11.900	0.003
x_1_	3.280	1	3.280	11.960	0.014
x_2_	0.218	1	0.218	0.795	0.407
x_3_	3.540	1	3.540	12.910	0.012
x_1_x_2_	1.250	1	1.250	4.560	0.077
x_1_x_3_	0.845	1	0.845	3.080	0.130
x_2_x_3_	5.640	1	5.640	20.600	0.004
x_1_^2^	2.710	1	2.710	9.900	0.020
x_2_^2^	0.669	1	0.669	2.440	0.169
x_3_^2^	0.669	1	0.669	2.440	0.169
x_1_x_2_x_3_	2.530	1	2.530	9.240	0.023
x_1_^2^ x_2_	0.610	1	0.610	2.230	0.186
x_1_^2^ x_3_	2.860	1	2.860	10.450	0.018
x_1_x_2_^2^	0.0504	1	0.0505	0.184	0.683
Residual	1.640	6	0.274	-	-
Lack of fit	0.569	1	0.569	2.650	0.165
Pure error	1.0800	5	0.215	-	-

### 3.4 Three dimensional plots

Fig. 1a plot showed that the two factors (acid concentration and temperature) have little significant effect when combined on the percentage yield. The effect of activation temperature is relatively higher than the effect of acid concentration as a result of their F- value. Increase in any of these two factors results in percentage yield increase. The effect activation temperature and acid concentration on Pb^2+^ uptake at constant activation time as shown in Fig. 1b revealed that the outcome is completely almost because of the singular impact of acid concentration with activation temperature having very minimal effect. The plot showed that removal efficiency of Pb^2+^ is increased appreciably with decrease in acid concentration, thus; rise in activation temperature results in generally very small increase in the removal of Pb^2+^. However, it is worthy to state that acid concentration increase past this limit will not result in any substantial change in the uptake capacity because further acid concentration increase may lead to clay mineral structural damage and as a result, there is bound to be reduction in the specific surface region. Hence, maximum removal of Pb^2+^is associated with minimum acid concentration. The effect of activation time and acid concentration as shown in Fig. 2a shows significant effect on the percentage yield based on their F- value with acid concentration showing more effect though activation time shows a reasonable effect too. Increase in acid concentration as revealed by the plot increases the percentage yield. However, increase in the acid concentration causes a decrease in the yield percent but with much effect at high activation time. The effect of acid concentration and activation time on percentage Pb^2+^ removal as seen in Fig. 2b, it was observed that decrease in acid concentration with activation time increase resulted to Pb^2+^ uptake increases. This indicates the fact that specific surface area, porosity and micro porosity of the activated clay were emphatically influenced by the activation time. Furthermore, maximum Pb^2+^ removal is associated with maximum activation time. Fig. 3a depicts that activation time and temperature at constant acid concentration have a considerable effect on the yield percentage. The plot observed that the effect of activation temperature is higher relatively to that of activation time and any of the two factors increase will reasonably leads to percentage yield increase. The effect of activation temperature and time at constant acid concentration on the percentage Pb^2+^ removal (see Fig. 3b) Plot revealed that the two parameters studied are almost completely as a result of the activation time singular effect with minimal effect from the activation temperature. It was additionally seen from the plot that increases in the activation time and temperature leads to percentage Pb^2+^ uptake increase since the textural properties and the adsorbent surface area rises with increase in activation temperature and time. Thus; at higher activation time (120 min) and temperature (100 °C) with low acid concentration (0.5 M), high surface area was achieved.

**Fig. 1:** Effect of acid concentration and temperature on percentage (a) yield and (b) Pb^2+^ removal on HCl activated Aloji clay (constant time = 75 min).

**Fig. 2:** Acid concentration and time effect on percentage (a) yield and (b) Pb^2+^ removal on HCl activated Aloji clay (constant activation temperature 85 °C).

**Fig. 3:** Effect of activation time and temperature on percentage (a) yield and (b) Pb^2+^ removal on HCl activated Aloji clay (constant acid activation = 2.25 M).

### 3.5 BET and FTIR analysis

Functional groups such as alumina, silicon and hydroxyl groups which are capable of adsorbing contaminants are mainly identified by FT-IR techniques. FT-IR spectra ranges from 500-4000 cm^−1^ wave number for raw and activated Aloji clay samples were characterized. To reflect the complex nature of the clay samples, a number of adsorption peaks were displayed and a few peaks were seen to have moved or vanished and new ones were detected after comparing the FT-IR analysis of raw to activated clay samples (see Fig. 4a and b). These observed change in the spectra of both clay samples confirmed that activation process modified the clay sample [22]. The untreated clay sample showed adsorption bands at 525, 602, 648, 756, 795, 918, 1034, and 1512 cm^−1^. However, after treatment with HCl, the new bands were formed at 3124, 3448, 3526 and 3618 cm^−1^ respectively and this was attributed to the Al– O– H stretching (physiosorbed water) while bands at 3649, 3695, 3742, 3865, 3896 and 3927 were attributed to Al– O– H stretching (structural hydroxyl groups and octahedral). The band vibrational at 1512 cm^−1^ related with H– O– H bending (physisorbed) was modified to 2932 cm^−1^ while band at 525 cm^−1^ relating to Si– O– Al stretching and 1034 cm^−1^ relating to the Si– O stretching remained after acid leaching. The bands at 602, 648, 687, 756, 795 and 918 cm^−1^ were completely absent after HCl activation [23, 24, 25, 26, 27].

**Fig. 4:** FT-IR result for (a) raw (b) HCl activation Aloji clay.

The BET result as summarized in Table 6 shows surface area, total pore volume and total pore size of untreated and activated Aloji clay. Untreated clay has surface area of 138.70 m^2^/g, pore volume of 0.0711 cm^2^/g and pore size of 1.17 nm. The surface area, pore volume and pore size further increased on activation with acid to 214.80 m^2^/g, 0.121 cm^2^/g and 1.43 nm. This increase can be attributed to the acid treatment of the clay as a result of exchangeable cations elimination and silica generation [21]. The raw and acid activated clay was established to be microporous (<2 nm) with pore average diameters of 1.17 and 1.43 nm respectively. The clay's (raw and activated clay) micropores presence could be attributed to the origin or the starting clay minerals type [28].

**Table 6:** BET analysis result for raw and acids activated Aloji clay.

Samples	Surface area (m^2^/g)	Pore volume (cc/g)	Pore size (nm)
Raw Aloji clay	138.70	0.0711	1.17
HCl activated Aloji clay	214.80	0.1210	1.43

### 3.6 Effect of initial Pb^2+^ concentration and time on adsorption

Pb^2+^ concentration and adsorption time effects under study on the quantity adsorbed are vital aspect of process adsorption. Initial concentation of Pb^2+^ varying from 30 to 150 mg/L were used to study adsorption capacity on acid activated clay (adsorbent). The results as depicted in Fig. 5 revealed that equilibrium was achieved slower (longer time) for higher concentrations and faster (shorter time) for those at lower concentrations. This could be as a result of the adsorbent having more vacant sites with minimal number of adsorbate molecules to adsorb thereby resulting in rapid adsorption available molecules (adsorbate). The attainment of equilibrium at longer time with higher concentration of Pb^2+^ can be accredited to the fact that: firstly, before saturation at constant adsorbent dosage, more molecules are waiting to be adsorbed at limited vacant sites thereby resulting in the adsorbent queue formation. Secondly, the series of adsorption processes which the adsorbates undergo are: molecules movement through a boundary layer to the external adsorbent surface and molecules diffusion into the adsorbent pores. Thirdly, adsorbates diffuse into adsorbent interior pores [9]. At 30 mg/L of Pb^2+^ concentration, equilibrium position was achieved after 30 min while at 60, 100 and 150 mg/L Pb^2+^ concentrations it took equilibrium position about 60 min to be established (Fig. 6). This is because more adsorbate molecules are in the aqueous solution challenging for the adsorbent available binding sites at a concentration higher than at lower concentrations thereby resulting in higher adsorption capacity [29].

**Fig. 5:** Initial concentration effect on the equilibrium removal of Pb^2+^ onto acid activated Aloji clay (temperature = 30 °C, rpm = 140, V = 100 ml, W = 0.10 g, pH 7).

**Fig. 6:** Adsorption time effect on the adsorption capacity of Pb^2+^ onto acid activated Aloji clay (temperature = 30 °C, rpm = 140, V = 100 ml, W = 0.10 g, pH 7).

### 3.7 Effect of adsorbent dosage

Adsorbent dosage effect was determined on Pb^2+^ adsorption uptake. The activated clay dosage (0.1–0.5 g) was varied with constant 100 mg/L Pb^2+^ concentration and 60 min (adsorption time) at 30 °C. The result as depicted in Fig. 7 revealed increases in the quantity of adsorbed Pb^2+^ with increasing adsorbent dosage. Adsorbent dosage (0.1–0.4 g) gives a faster increase in the Pb^2+^ percentage removal while further adsorbent dosage increase beyond this point (0.5 g) did give a satisfactory increase in the Pb^2+^ uptake due to the unavailability of more vacant site for adsorption. This result also indicated that at lower adsorption dosage with limiting adsorption sites, metal ions compete for adsorption. Accessibility of adsorption sites advances adsorption which results in a more prominent removal of Pb^2+^ as the quantity of adsorbent dosage is increased [30].

**Fig. 7:** Adsorbent dosage effect on Pb^2+^ adsorption for HCl activated Aloji clay (Time = 60 min, Temperature = 30 °C, V = 100 mL and initial Concentration = 100 mg/L, pH 7).

### 3.8 Adsorption isotherm

#### 3.8.1 Langmuir isotherm

Langmuir adsorption isotherm linearized form is given as: [31].

(7) $$\frac{{\text{C}}_{\text{e}}}{{\text{q}}_{\text{e}}}=\frac{1}{{\text{q}}_{\text{max}}{\text{K}}_{\text{L}}}+\frac{{\text{C}}_{\text{e}}}{{\text{q}}_{\text{max}}}$$

C_e_ is the adsorbate concentration at equilibrium (mg/L), q_e_ is the quantity of Pb^2+^ adsorbed (mg/g), q_max_ and K_L_ (Langmuir constant), the monolayer adsorption capacity and adsorbent-adsorbate affinity respectively. The graph of ceqe is plotted against C_e._ The dimensionless constant R_L_ was used to ascertain the Langmuir model fitness and the values obtained are interpreted as follows: R_L_> 1 (unfavorable), 0 < R_L_< 1 (favorable), R_L_ = 1 (linear) or R_L_ = 0 (irreversible). The dimensionless factor R_L_ equation is given as: [32].

(8) $$R_{L}=\frac{1}{1+{\text{K}}_{\text{L}}{\text{C}}_{\text{o}}}$$

${\text{K}}_{\text{L ​}}$ is Langmuir constant and C_o_ is the highest concentration of Pb^2+^ (mg/L).

#### 3.8.2 Freundlich isotherm

The Freundlich isotherm model linearized form is given by [33]:

(9) $${\text{logq}}_{\text{e}}={\text{ ​log ​k}}_{\text{f}}+\frac{1}{\text{n}}{\text{log ​C}}_{\text{e}}$$

q_e_ is quantity adsorbed at equilibrium (mg/g), C_e_ is the adsorbate equilibrium concentration (mg/L), k_f_ (l/g) and n are the Freundlich equilibrium coefficients. The n values give favourability information of the adsorption process while k_f_ is the adsorbate adsorption capacity.

The graph of log q_e_ is plotted against log C_e_

#### 3.8.3 Temkin isotherm

The Temkin model isotherm linearized form is given by [34].

(10) $${\text{q}}_{\text{e ​}}=B\;\ln\;{\text{A}}_{\text{T}}+B\;\ln\;{\text{C}}_{\text{e}}$$

Where A_T_ is the equilibrium binding constant, B is the adsorption heat, q_e_ is the adsorption capacity (mg/g) and C_e_ is the equilibrium concentration of adsorbed Pb^2+^ (mg/L).

(11) $$B=\frac{\text{RT}}{{\text{b}}_{\text{T}}}$$

$\frac{1}{{\text{b}}_{\text{T}}}$ Indicated the adsorption potential of the adsorbent, R is the universal gas constant (8.314 J/kmol) and T is the temperature (K). The graph of q_e_ is plotted against$\text{ ​ln}C_{e}$at various temperatures.

Langmuir, Freundlich and Temkin isotherms study in this research work described the Pb^2+^ adsorption on activated clay with fitness consideration on some level of variance. Adsorption isotherms with best fit (closest to 1) based on the highest correlation coefficient (R^2^) value was selected and this helps to describe the fitness of isotherms to the experimental data. Among other isotherm models studied, Freundlich model had the best fit (Fig. not shown); as evidented in the R^2^ values summarized in Table 7 and Fig. 8. Results also showed Langmuir and Temkin models as second and third after Freundlich model, respectively. Furthermore, best fit of Freundlich model to the adsorption process which goes by the informed values of n > 1 and 0 < 1/n < 1 obtained, satisfies both favourability and surface heterogeneity of the adsorption surface of activated Aloji clay with values between 0 and 1 and becoming more heterogeneous as the values decreases (tends to 0) [29]. Although, Langmuir isotherm was the second fitted model, favourable adsorption of Pb^2+^ on the homogeneous surface of the activated Aloji clay was observed; this is going by the range of values obtained from 0.010-0.072 satisfying the condition 0 < R_L_ < 1. The predicted maximum adsorption capacity from the Langmuir model increased from 166.667 to 333.333 mg/g for an increase temperature from 30 to 50 °C. Temkin isotherm assumed that coverage increase leads to decrease in heat adsorption of all molecules layer due to solid-liquid interaction and that binding energies are characterized by homogeneous distribution [9, 30]. Table 8 shows the comparison of monolayer adsorption of Pb^2+^onto various adsorbent.

**Table 7:** Langmuir, Freundlich and Temkin models for Pb^2+^ on HCl activated Aloji clay.

Isotherms	Parameters	30 °C	40 °C	50 °C
Langmuir	q_m_(mg/g)	166.667	250.000	333.333
	K_L_ (L/g)	0.667	0.586	0.428
	R^2^	0.941	0.946	0.958
Freundlich	k_f_	74.645	83.560	84.528
	1/n	0.299	0.261	0.223
	R^2^	0.998	0.999	0.999
Temkin	A_T_ (L/mg)	69.598	169.917	516.134
	b_T_ (KJ/mol)	124.035	141.428	176.905
	R^2^	0.841	0.847	0.922

**Fig. 8:** Plots for (a) Langmuir, (b) Freudlich and (c) Temkin isotherms for Pb^2+^ adsorption on acid activated Aloji clay at 30 °C.

**Table 8:** Sorption capacities of lead ions by natural and synthetic adsorbents.

Adsorbent	Maximum adsorption capacity (mg/g)	References
Bentonite clay	28.00	[35]
Kaolinite clay	31.75	[36]
Illite clay	25.44	[37]
KC clay	86.40	[38]
Zeolite	24.40	[39]
Paper sludge	103.50	[40]
Montmorillonite clay	37.16	[41]
Zeolite- Kaolin- Bentonite	108.70	[42]
Turkish illite clay	238.98	[43]
Polyaniline/montmorillonite composite	308.60	[44]
HCl activated Aloji clay	333.33	Present work

### 3.9 Adsorption kinetics models

#### 3.9.1 Pseudo-first order model

The pseudo-first order kinetic linearized form is given by [45].

(12) $$\log\text{ ​}\left({\text{q}}_{\text{e ​}-}{\text{q}}_{\text{t}}\right)=\log\;{\text{q}}_{\text{e ​}-}\frac{{\text{k}}_{1}\text{t}}{2.303}$$

q_e_ and q_t_ are the quantity of Pb^2+^ adsorbed at equilibrium and time t(h) respectively, (mg/g). k_1_ is adsorption rate constant (min^−1^). The graph of$\text{ ​ ​log}\;(q_{e-}q_{t}$) is plotted against t at different temperatures studies.

#### 3.9.2 Pseudo-second order model

The pseudo-second order model linearized form is given by [46].

(13) $$\frac{\text{t}}{{\text{q}}_{\text{t}}}=\frac{\text{t}}{{\text{q}}_{\text{e}}}+\frac{1}{{\text{k}}_{2}{\text{q}}_{\text{e}}^{2}}$$

k_2_ (g/mgmin) is the adsorption rate constant. The graph of $\frac{t}{q_{t}}$ versus t is plotted at different temperatures studies.

The adsorption kinetic models result showed that both models studied described the process adsorption but, the best description was given by pseudo-second-order as depicted in Table 9 and Fig. 9 when compared. The pseudo-second order adsorption rate constant (k_2_) is smaller and decreases when compared with that of pseudo-first order (k_1_) indicating that adsorption takes place faster at lower concentration. However, the values of adsorption capacity (q_e_cal) calculated for Pseudo-second order were seen to be more close to the adsorption capacity of the experimental values (q_e_exp) to those of the pseudo-first-order. Furthermore, the R^2^ correlation coefficient values of the pseudo-second order were more tending to towards 1 (unity) than those of the pseudo-first order. Thus, the inability of the kinetics data fitness of the pseudo-first order could be attributed to the boundary layers limitations which control the sorption processes [47].

**Table 9:** Pseudo-first and second order kinetics for Pb^2+^ adsorption on HCl activated Aloji clay at 30 °C.

			Pseudo- first order			Pseudo- second order		
Adsorbents	Pb^2+^ conc. (mg/L)	q_e_exp (mg/g)	q_e_cal (mg/g)	k_1_ (min^−1^)	R^2^	q_e_cal (mg/g)	k_2_ (min^−1^)	R^2^
HCl activated Aloji Clay	30	28.36	8.810	0.0230	0.607	29.412	0.0170	0.999
	60	57.40	17.620	0.0300	0.661	58.824	0.00876	0.999
	100	95.40	42.170	0.0368	0.851	100.000	0.00345	0.998
	150	138.50	55.463	0.0415	0.830	142.857	0.00258	0.998

**Fig. 9:** Plots of (a) pseudo-first-order, (b) pseudo-second-order kinetics for Pb^2+^ on HCl activated Aloji clay at 30 °C.

### 3.10 Adsorption thermodynamics studies

Thermodynamic parameters for Pb^2+^adsorption on activated clay at various temperatures of 30, 40 and 50 °C were evaluated for process adsorption spontaneity. The thermodynamic equation is given as:

(14) $$\text{log ​}\frac{{\text{q}}_{\text{e}}}{{\text{C}}_{\text{e}}}=-\frac{\Delta {\text{H}}^{\text{O}}}{2.303\text{R}}(\frac{1}{T})+\frac{\Delta {\text{S}}^{\text{O}}}{2.303\text{R}}$$

R (8.314 J/kmol) universal constant, T is the absolute temperature (K), ΔH^o^ is the enthalpy change and ΔS is the entropy change. A Plot of$\;\text{log ​}\frac{q_{e}}{C_{e}}$ against $\frac{\;1}{T}$. The free Gibbs energy (ΔG^o^) is obtained using this equation:

(15) ΔG^o^ = ΔH^o^ -TΔS^o^

The thermodynamic result as depicted in Table 10 for Pb^2+^ adsorption onto activated Aloji clay (adsorbent) affirm to the spontaneous nature of the process adsorption as seen in the negative values of the Gibb's free energy (ΔG^o^). The enthalpy (ΔH^o^) positive values shows that the process is endothermic while positive entropy (ΔS^0^) values also revealed affinity and increase in randomness (degree of freedom) at the adsorbent-adsorbate boundary during process adsorption [48, 49]. The absolute value change of Gibbs free energy for physical adsorption is −20 to 0 kJ/mol and that of chemisorptions−80 to −400 kJ/mol [50]. The Gibbs free energy (ΔG^o^) result of this study affirmed that the nature of adsorption process is physical and involves attraction of weak forces at the adsorbate-adsorbent interface [48, 51].

**Table 10:** Thermodynamics parameters of Pb^2+^ adsorption on HCl activated Aloji clay at 150 mg/L.

Adsorbate	Pb^2+^ conc. (mg/L)	ΔH^o^ (kJ/mol)	ΔS^o^ (J/Kmol)		ΔG^o^ (kJ/mol)		R^2^
Pb^2+^				30 °C	40 °C	50 °C	
	150	4.808	40.018	-7.318	-7.718	-8.117	0.993

## 4 Conclusions

A batch process adsorption Pb^2+^ uptake from aqueous solution onto modified Aloji clay as an adsorbent was carried out. Central composite design (CCD) was used to optimized Aloji clay modification at different variables which are; activation temperature, activation time and acid concentration with yield percentage and Pb^2+^ as the responses under study. Optimal condition of 0.5 M, 100 °C and 120 min translated into 55.65 and 97.33 % for yield and Pb^2+^ removal. The effect Pb^2+^ concentration, adsorbent dosage, temperature effect and adsorbent time were all examined with equilibrium attainment of the adsorption process at 60 min. The activated Aloji clay BET specific surface area of 214.80 m^2^/g, cumulative pore volume of 0.121 cm^3^/g and an average pore diameter of 1.43 nm resulted into maximum monolayer capacity of 333.333 mg/g. The isotherm model studied showed Freundlich model as the best fit followed by Langmuir and Temkin, respectively. The adsorption of Pb^2+^ onto activated Aloji clay as revealed by the thermodynamics studies is endothermic, spontaneous, physical in nature and it obey's pseudo-second-order kinetics. This study showed that Aloji clay has the effective and efficient potential to be use for as replacement for expensive absorbent for Pb^2+^ uptake from aqueous solutions.

## Declarations

### Author contribution statement

Auta Manase: Conceived and designed the experiments.

Shola Obayomi: Performed the experiments; Analyzed and interpreted the data; Contributed reagents, materials, analysis tools or data; Wrote the paper.

### Funding statement

This research did not receive any specific grant from funding agencies in the public, commercial, or not-for-profit sectors.

### Competing interest statement

The authors declare no conflict of interest.

### Additional information

No additional information is available for this paper.
